# Risk Factors and Prediction Models for Nonalcoholic Fatty Liver Disease Based on Random Forest

**DOI:** 10.1155/2022/8793659

**Published:** 2022-08-09

**Authors:** Qingqun Li, Xiuli Zhang, Chuxin Zhang, Ying Li, Shaorong Zhang

**Affiliations:** Shengzhen (Guangming) Hospital, University of Chinese Academy of Sciences, Shenzhen 230031, China

## Abstract

**Objective:**

To establish a risk prediction model of nonalcoholic fatty liver disease (NAFLD) and provide management strategies for preventing this disease.

**Methods:**

A total of 200 inpatients and physical examinees were collected from the Department of Gastroenterology and Endocrinology and Physical Examination Center. The data of physical examination, laboratory examination, and abdominal ultrasound examination were collected. All subjects were randomly divided into a training set (70%) and a verification set (30%). A random forest (RF) prediction model is constructed to predict the occurrence risk of NAFLD. The receiver operating characteristic (ROC) curve is used to verify the prediction effect of the prediction models.

**Results:**

The number of NAFLD patients was 44 out of 200 enrolled patients, and the cumulative incidence rate was 22%. The prediction models showed that BMI, TG, HDL-C, LDL-C, ALT, SUA, and MTTP mutations were independent influencing factors of NAFLD, all of which has statistical significance (*P* < 0.05). The area under curve (AUC) of logistic regression and the RF model was 0.940 (95% CI: 0.870~0.987) and 0.945 (95% CI: 0.899~0.994), respectively.

**Conclusion:**

This study established a prediction model of NAFLD occurrence risk based on the RF, which has a good prediction value.

## 1. Introduction

Nonalcoholic fatty liver disease (NAFLD) is a metabolic stress liver injury closely related to insulin resistance and genetic susceptibility. Its pathological changes are similar to those of alcoholic liver disease, but the patient has no history of excessive drinking [1]. The spectrum of diseases includes nonalcoholic simple fatty liver, nonalcoholic steatohepatitis, and hepatocellular carcinoma [2, 3]. With the continuous improvement of people's living standards, the traditional diet structure in China has also changed. The prevalence of NAFLD has increased significantly, becoming a severe health problem. Studies have shown that the prevalence of NAFLD among the global general population is 6.3%-45% [4], and the probability of other diseases is as high as 58.9%. NAFLD has become a major liver disease in Europe's developed and economically developed areas [5, 6]. In China, with the increase in obesity, diabetes, and hyperlipidemia, NAFLD has surpassed viral hepatitis and alcoholic liver disease and has become the leading cause of chronic liver disease in China [7]. With the prevalence of obesity and metabolic syndrome, NAFLD has become China's most prominent chronic liver disease. It is also the primary cause of abnormal liver enzymes in physical examination, which seriously endangers people's lives and health [8]. NAFLD has become not only a global disease but also a social issue of universal concern [9].

The pathogenesis of NAFLD is still unclear, involving many factors such as heredity, environment, and lifestyle. It is related to obesity, gender, hyperlipidemia, insulin resistance, and diabetes. Thus, it can be considered a metabolic syndrome component [10, 11]. Studies have shown that insulin resistance and lipid metabolism disorder are the central links in the pathogenesis of NAFLD. The corresponding hyperinsulinemia and hyperlipidemia increase the toxicity of glucose and fat, thus causing liver damage. In addition, the body produces metabolic stress reaction, which leads to metabolic dysfunction [12, 13]. Metabolic syndrome is a clinical syndrome in which obesity, impaired glucose tolerance, lipid metabolism disorder, hypertension, hyperuricemia, and other risk factors are concentrated in the same body [14, 15]. In addition, microsomal triglyceride transfer protein (MTTP) exists in hepatocytes, and the polymorphism of the MTTP gene is related to its gene activity [16]. Liver steatosis and fibrosis are more common in patients with low active genotype fatty liver, suggesting that MTTP gene polymorphism may affect the course of fatty liver [17, 18].

In recent years, machine learning based on random forest (RF) and other algorithm have been widely applied in the medical field [19–23]. Therefore, this study is aimed at establishing a risk prediction model of NAFLD based on routine physical examination indexes through a retrospective cohort study and at providing new ideas for the early identification of high-risk groups of NAFLD patients. In addition, the analysis of disease gene polymorphism has also opened up a brand-new field for exploring the diversification of clinical phenotype and individualized clinical treatment of NAFLD.

## 2. Materials and Methods

### 2.1. Research Object

From June to December 2020, 200 inpatients and physical examinees were collected from the Department of Gastroenterology and Endocrinology and Physical Examination Center of Shenzhen Hospital of the Chinese Academy of Sciences. There is no blood relationship between the subjects, all of whom are Han people in Guangming District. An informed consent form was signed with the consent of the Ethics Committee of Shenzhen Hospital of the University of Chinese Academy of Sciences.

### 2.2. Inclusion Criteria

Inclusive criteria included clinical diagnostic criteria and B-ultrasound results. Among them, the clinical diagnostic criteria include the following: (1) no history of drinking or alcohol consumption is less than 140 g per week for men and less than 70 g per week for women; (2) except for viral hepatitis, drug-induced liver disease, total parenteral nutrition, hepatolenticular degeneration, autoimmune liver disease, and other specific diseases that can lead to fatty liver; and (3) histological changes of liver biopsy conform to the pathological diagnostic criteria of fatty liver venereal disease. Because of the difficulty in obtaining a histological diagnosis of the liver, NAFLD work is defined as that the imaging findings of the liver meet the diagnostic criteria of diffuse fatty liver without other reasons to explain. And (or) patients with metabolic syndrome-related components have unexplained serum alanine aminotransferase (ALT) and (or) aspartate transaminase (AST) and *γ*-glutamine transferase (GGT) continuously increased for more than half a year. After losing weight and improving insulin resistance, the diagnosis of NAFLD can be confirmed if an abnormal zymogram and imaging fatty liver are improved or even returned to normal.

In addition, two of the following four abdominal ultrasounds are diffuse fatty liver: (1) the near-field echo of the liver area is diffusely enhanced, and the echo is stronger than that of a kidney. (2) The far-field echo gradually attenuates. (3) The intrahepatic duct is not displayed. (4) The liver may be slightly or moderately enlarged.

### 2.3. Exclusion Criteria

Exclusion criteria include (1) long-term drinking history, less than 210 g in a week for men and less than 140 g in a week for women; (2) fatty liver caused by viral hepatitis, drug-induced liver disease, total parenteral nutrition, hepatolenticular degeneration, autoimmune liver disease, etc.; (3) pregnant and lactating women; and (4) anyone who has taken any drugs that affect sugar and lipid metabolism and blood pressure in the last month.

### 2.4. Collection of Clinical Data and Laboratory Examination Indexes

The gender, age, waist circumference (WC), BMI, systolic blood pressure (SBP), and diastolic blood pressure (DBP) were measured. After fasting for 12 hours, all the above-mentioned people collected fasting venous blood the next morning, and some of them were used for whole blood DNA extraction. The laboratory indexes include fasting plasma glucose (FPG), total cholesterol (TC), triglyceride (TG), high-density lipoprotein cholesterol (HDL-C), low-density lipoprotein cholesterol (LDL-C), ALT, AST, GGT, and uric acid (UA). In addition, we also detected the gene of the MTTP. The PCR product after partial purification of the MTTP gene was sequenced to screen out the mutant gene.

### 2.5. Data Preprocessing

Because the original data set extracted from the database may contain some problems such as missing values, abnormal values, or uneven sampling, data modeling cannot be done directly. Therefore, it is necessary to preprocess the original data set. The specific process is shown in Figure 1. Firstly, data set labeling is carried out, the main purpose of which is to supplement the collected case data with corresponding labels as the gold standard for training and testing machine learning algorithms. In this paper, according to the ultrasonic image examination report results, cases with diagnosed fatty liver are identified as 1, and cases without fatty liver are identified as 0. Then, the data is cleaned to check whether there are missing values, redundant contents (duplicate data and irrelevant data), and noisy data (erroneous data and abnormal data). Finally, standardize the data. In order to eliminate the influence of dimensional differences among different features (independent variables), it is necessary to standardize the data.

This study adopts zero-mean normalization (also called Z-score normalization). The mean value of the processed data is 0 and the standard deviation is 1. The calculation formula is

(1) $$\begin{array}{c} x^{\prime }=\frac{x-\mu }{\sigma }. \end{array}$$

After zero-mean normalization, the original data conform to the standard normal distribution. The standard partial regression coefficient is calculated according to the normalized data set. The greater the absolute value of the coefficient, the greater the influence of the independent variable on the dependent variable.

### 2.6. Construction of Random Forest Prediction Model

Random forest refers to a classifier that uses multiple trees to train and predict samples, which belongs to an integrated algorithm. The application effect of RF in classification, regression, and clustering is good [24]. Assuming that there are *M* samples and *n* feature data sets, at most, *t* decision trees must be constructed, and the number of features in each decision tree is *K*; then, the realization process of the RF algorithm is as follows:

(2) $$\begin{array}{c} f\left(x\right)=\begin{array}{c} \min\\ j,s \end{array}\left[\begin{array}{c} \min\\ c_{1} \end{array}\underset{x_{i}\in R_{1}\left(j,s\right)}{\sum }{\left(y_{i}-c_{1}\right)}^{2}+\begin{array}{c} \min\\ c_{2} \end{array}\underset{x_{i}\in R_{2}\left(j,s\right)}{\sum }{\left(y_{i}-c_{2}\right)}^{2}\right]. \end{array}$$

*R*_1_ and *R*_2_ represent the divided two subsets (regression tree is a binary tree with only two subsets). *c*_1_ and *c*_2_ represent the average values of *R*_1_ and *R*_2_ samples, respectively. *J* represents the characteristics of the sample, *s* represents the dividing point, and *y*_*i*_ represents the true value of the target variable of the sample. Use the selected (*j*, *s*) to divide the area and determine the corresponding output value. The formula for finding the sample mean is

(3) $$\begin{array}{c} {\hat{c}}_{m}=\frac{1}{N_{m}}\underset{x_{i}\in R_{1}\left(j,s\right)}{\sum }y_{i}. \end{array}$$

Divide the input sample into *m* regions, namely, *R*_1_, *R*_2_, ⋯, *R*_*m*_ to generate the decision tree. The formula is as follows:

(4) $$\begin{array}{c} f\left(x\right)=\overset{M}{\underset{m=1}{\sum }}{\hat{c}}_{m}I. \end{array}$$

*C* represents the average value of the corresponding area, and *I* represents whether it meets the conditions. If it meets the conditions, it is 1; otherwise, it is 0.

By sampling with replacement, a data set with *M* samples is obtained from the original data set through *M* sampling times. From the *n* features, the principle of no-replacement sampling is adopted, and *K* features are removed as input features. Repeat the above process *t* times for the new data set to build *t* decision trees. Average the generated *t* decision trees, and finally, get a random forest model (Figure 2).

The overall data processing flow based on machine learning is shown in Figure 3. All the research indicators are added to the experimental data set and used as training sets to train common machine learning algorithm models. The specific method is to randomly select 70% of the preprocessed physical examination data of 200 cases as the training set (*n* = 140) and the remaining 30% as the verification set (*n* = 60). Then, the prediction performance of the RF machine learning model is evaluated by using the 50% cross-validation method and repeating the experiment 10 times and averaging the results.

### 2.7. Statistical Analysis

The SPSS23.0 software was used for data analysis. All data are expressed as $\overset{¯}{x}\pm s$. The measurement data conforms to the two groups' normal distribution, and the *t*-test is adopted. Nonparametric statistics are used after the variance homogeneity test for nonnormal distribution. The data were counted by the chi-square test. Logistic regression analysis was used for multiple regression analysis of risk factors. *P* < 0.05 is considered to be statistically significant.

## 3. Results

### 3.1. Comparison of Research Variables

A total of 200 subjects were included in this study, including 140 in the training set and 60 in the verification set. A total of 44 patients developed NAFLD, and the cumulative incidence rate was 22%. Among them, the number of NAFLD patients in the training set is 31 and the cumulative incidence rate is 22.1%. The number of patients with NAFLD in the validation set was 13 and the cumulative incidence rate was 21.7%. There was no significant difference in sex, age, WC, BMI, SBP, DBP, FPG, TG, TC, HDL-C, LDL-C, ALT, AST, GGT, SUA, WBC, NLR, MTTP, MTTP mutations, and the incidence of NAFLD between the training set and the verification set (*P* > 0.05). The two sets of data are comparable (Table 1).

### 3.2. Logistic Regression Risk Prediction Model

Multivariate logistic regression analysis was used to analyze the independent risk factors of NAFLD, and 16 variables with statistical significance after single factor analysis were included in the analysis. Then, all the meaningful indicators of single-factor analysis results are brought into the one-way variance analysis. The results showed that BMI, TG, HDL-C, LDL-C, ALT, SUA, and MTTP mutations were independent influencing factors of NAFLD, all of which had statistical significance (*P* < 0.05) (Table 2).

### 3.3. Random Forest Risk Prediction Model

The RF is an ensemble learning method based on a decision tree as the basic classifier, random attribute selection is introduced in the training process, and the final classification result is obtained by voting through multiple decision trees. The ranking results of independent variables comprehensively scored based on the stochastic forest prediction model are shown in Figure 4.

### 3.4. Evaluation of NAFLD Occurrence Risk Prediction Model

The receiver operating characteristic (ROC) curve was used to verify the established NAFLD occurrence risk model. The results showed that the area under the curve (AUC) of the logistic regression model was 0.940 (95% CI: 0.870~0.987) and that of RF was 0.945 (95% CI: 0.899~0.994) in the training set (Figure 5).

## 4. Discussion

As a metabolic disease involving multiple systems, NAFLD is closely related to the high incidence of extrahepatic malignant tumors such as cirrhosis, coronary heart disease, and chronic kidney disease [25]. The prevalence of NAFLD has become a new challenge in public health and poses a serious threat to people's health and safety [8, 26]. The pathogenesis of NAFLD is not clear. Viral infection, autoimmune liver disease, oxidative stress, insulin resistance, heredity, and intestinal flora disorder can all lead to this disease [10]. More and more research is being paid to exploring the influencing factors of NAFLD, building a crowd risk prediction model, identifying high-risk groups, and diagnosing and preventing NAFLD in advance [19]. Therefore, a good prediction model will accurately predict the progress of the disease, so as to effectively monitor and timely intervene the high-risk groups. Therefore, it is the key to establish the forecasting model to select easily available and accurate prediction indicators.

In this study, based on random forest and logistic regression, a prediction model of NAFLD risk was constructed, which included 15 indexes such as physical examination, laboratory examination, and gene screening. The results showed that high BMI and age were independent risk factors for NAFLD, which is consistent with previous studies involved in the establishment NAFLD risk model [26, 27]. This result may be related to the low level of physical activity. An investigation shows that sedentary behavior is positively correlated with NAFLD [28]. A recent cross-sectional study on young people confirmed that physical activity was independently related to the degree of hepatocytes damage and the risk of NAFLD in the general population [29]. As an independent risk factor of NAFLD, UA also participated in the construction of the NAFLD risk model in this study. The reason is that UA can increase insulin resistance sensitivity and induce NAFLD. Hyperuricemia can stimulate oxidative stress in mitochondria and endoplasmic reticulum and induce lipid biosynthesis in hepatocytes [30]. Therefore, UA-lowering therapy may become an effective way to prevent NAFLD. The liver mainly produces serum GGT, so it can reflect the synthesis and reserve ability of the liver and can also be used to assess the degree of liver parenchymal cell injury by testing [31]. When hepatocytes are damaged, the pressure in the bile duct will rise, thus affecting bile excretion function, and the GGT level will also increase significantly.

Previous studies have shown that dyslipidemia is the key factor in the development of NAFLD [25]. The results show that TG and LDL-C are independent risk factors for NAFLD, and HDL-C is a protective factor for NAFLD. Many studies have confirmed that the excessive accumulation of lipids intensifies the production of reactive oxygen species, which destroys the steady state of redox by inducing oxidative stress and activates the inflammatory signal-mediated proinflammatory reaction, thus causing further damage to the hepatocytes [32, 33]. In addition, high TG can cause insulin resistance, leading to hyperglycemia. Elevated blood sugar will stimulate insulin secretion, which in turn will promote the synthesis of TG and LDL-C in hepatocytes, forming a vicious circle, resulting in lipid accumulation in hepatocytes [34]. ALT is an important catalytic enzyme in the human body, mainly in hepatocytes. The results of this study confirm that ALT can be used as a predictive index for the new occurrence of NAFLD. A recent study demonstrated that high ALT levels can reduce insulin sensitivity in hepatocytes, further affect glucose levels and fat accumulation in the human body, and aggravate the occurrence and development of NAFLD [35].

In addition, the polymorphism of the MTTP gene was also studied. MTTP transports fat out of the liver, so the lipid excretion from the liver is affected by the change in MTTP [36]. The G/T polymorphism at the -493 site of the MTTP promoter region is related to low-level transcription, which can result in the decrease in MTTP. TG could not be excreted from the liver, which promotes the pathogenesis of NAFLD [37]. This study confirmed that the mutation rate of MTTP gene in patients with NAFLD was high, which is similar to previous studies [38].

To predict the effectiveness of the prediction model, the ROC curve analysis was carried out in this study. The results showed that the AUC of the logistic regression model was 0.940 (95% CI: 0.870~0.987) and that of RF was 0.945 (95% CI: 0.899~0.994) in the training set. It is suggested that the prediction model is valuable for predicting the risk of NAFLD and is of great significance for clinical screening of patients with NAFLD.

## 5. Conclusions

To sum up, based on the RF algorithm, this study established a prediction model of NAFLD occurrence risk, which has good prediction value. As the number of cases selected in this study is small and the data used are from a single center, it is necessary to construct a prediction model based on a long-term follow-up survey of more samples and carry out effective external verification, to provide an important reference value for clinical screening of NAFLD risk factors.

## Figures and Tables

**Figure 1:** Data set preprocessing process.

**Figure 2:** Flow chart of random forest construction.

**Figure 3:** Data processing process based on machine learning.

**Figure 4:** Importance rating of characteristic variables based on random forest.

**Figure 5:** ROC curves obtained by the prediction models based on logistic regression and random forest.

**Table 1:** General data comparison between training set and verification set.

Variable	Training set	Validation set	*t*/*x^2^*/Z	*P*
Gender (male/female)	60/80	17/43	3.742	0.053
Age (years)	39.1 ± 9.34	39.2 ± 9.41	0.069	0.945
WC (cm)	79.56 ± 9.28	79.48 ± 9.32	-0.056	0.956
BMI (kg/m^2^)	23.15 ± 2.36	23.21 ± 2.24	0.167	0.867
SBP (mmHg)	123.26 ± 16.32	121.35 ± 15.68	-0.767	0.444
DBP (mmHg)	76.48 ± 10.36	75.89 ± 10.43	-0.368	0.713
NAFLD (%)	31 (22.1%)	13 (21.7%)	0.006	0.941
FPG (mmol/L)	5.30 (5.00-5.61)	5.34 (5.01-5.62)	1.832	0.067
TC (mmol/L)	4.84 ± 0.94	4.86 ± 0.92	0.139	0.890
TG (mmol/L)	0.95 (0.71-1.36)	0.95 (0.72-1.38)	0.552	0.581
HDL-C (mmol/L)	1.35 ± 0.31	1.36 ± 0.30	0.211	0.833
LDL-C (mmol/L)	2.52 ± 0.68	2.51 ± 0.66	-0.096	0.924
ALT (U/L)	17.01 (13.11-23.53)	17.01 (13.15-23.56)	0.238	0.812
AST (U/L)	19.03 (16.10-22.23)	19.03 (16.08-22.23)	0.029	0.977
GGT (U/L)	15.00 (11.02-21.45)	15.00 (11.00-23.30)	0.985	0.325
UA (umol/L)	314.15 ± 79.56	312.36 ± 80.49	-0.145	0.885
MTTP mutations	25 (17.9%)	11 (18.3%)	0.006	0.936

**Table 2:** Multivariate logistic regression analysis of NAFLD risk in training set.

Variable	*β*	$S\bar{x}$	Wald *x*^2^	*HR* (95% *CI*)	*P*
BMI	0.198	0.023	90.564	1.219 (1.170~1.273)	<0.01
TG	0.113	0.032	13.846	1.116 (1.050~1.183)	<0.01
HDL-C	-1.087	0.316	20.982	0.332 (0.205~0.536)	<0.01
LDL-C	0.214	0.079	6.538	1.250 (1.050~1.491)	<0.05
ALT	0.016	0.005	11.195	1.015 (1.006~1.025)	<0.05
UA	0.005	0.003	12.184	1.004 (1.001~1.005)	<0.01
MTTP	0.997	0.056	8.671	2.71 (1.38~5.27)	<0.05

## Data Availability

The data used to support the findings of this study are available from the corresponding author upon request.
